This article has been retracted.

# Resveratrol Preincubation Enhances the Therapeutic Efficacy of hUC-MSCs by Improving Cell Migration and Modulating Neuroinflammation Mediated by MAPK Signaling in a Mouse Model of Alzheimer’s Disease

**DOI:** 10.3389/fncel.2020.00062

**Published:** 2020-03-27

**Authors:** Xinxin Wang, Junwei Wu, Shanshan Ma, Ya Xie, Hongtao Liu, Minghao Yao, Yanting Zhang, Greta Luyuan Yang, Bo Yang, Ruixia Guo, Fangxia Guan

**Affiliations:** ^1^Department of Gynecology, The First Affiliated Hospital of Zhengzhou University, Zhengzhou, China; ^2^Department of Urology, The First Affiliated Hospital of Zhengzhou University, Zhengzhou, China; ^3^School of Life Sciences, Zhengzhou University, Zhengzhou, China; ^4^Stuyvesant High School, New York, NY, United States; ^5^Department of Neurosurgery, The First Affiliated Hospital of Zhengzhou University, Zhengzhou, China; ^6^Institute of Stem Cell and Regenerative Medicine, The First Affiliated Hospital of Zhengzhou University, Zhengzhou, China

**Keywords:** Alzheimer’s disease, human umbilical cord-derived mesenchymal stem cells, resveratrol, MAPK, neuroinflammation

## Abstract

Human umbilical cord-derived mesenchymal stem cells (hUC-MSCs) are promising for the treatment of Alzheimer’s disease (AD). However, their low rate of migration and survival in the brain limit their clinical applicability. This study is designed to improve the therapeutic potential of hUC-MSCs by preincubating them with resveratrol, a natural polyphenol capable of regulating cell destiny. Herein, we demonstrate that resveratrol preincubation enhances the migration of hUC-MSCs *in vitro*, as well as their survival and homing into the hippocampus of AD mice *in vivo*. Moreover, resveratrol-primed MSCs were better able to inhibit amyloid-β peptide (Aβ) deposition, Tau hyperphosphorylation, and oxidative stress, all while improving learning and memory. Notably, we found that hUC-MSCs inhibited neuroinflammation by reacting with astrocytes and microglial cells and suppressing mitogen-activated protein kinases (MAPKs), extracellular signal kinases (ERK), p38 kinases (p38), and c-Jun N-terminal kinases (JNK) signaling pathways in the hippocampus of AD mice. Furthermore, resveratrol pretreatment enhanced these effects. Conclusively, the current study revealed that resveratrol preconditioning protected hUC-MSCs against the hostile microenvironment characteristic of AD and enhanced their viability and homing into the brain of AD mice. The use of resveratrol-pretreated hUC-MSCs is thereby proposed to be a promising therapy for AD.

## Introduction

Alzheimer’s disease (AD) is a devastating neurodegenerative disease. However, its pathogenesis and an effective treatment have yet to be further elucidated. In addition to extracellular deposition of amyloid-β peptides (Aβ) and intracellular aggregation of hyperphosphorylated tau, a number of studies have revealed that neuroinflammation is a critical event in the pathogenesis of AD (McGeer et al., 2016). Microglia and astrocytes are major cells involved in neuroinflammation. Upon activation, they can release proinflammatory cytokines, chemokines, neurotoxins, and reactive oxygen species (ROS), leading to chronic progressive neurodegeneration (Calsolaro and Edison, 2016). Thus, targeting the neuroinflammation caused by microglia and astrocytes represents a promising therapeutic strategy for AD.

Mesenchymal stem cells (MSCs) are multifunctional cells derived from bone marrow, adipose tissue, endometrium, the umbilical cord, and amniotic membrane, among others. Human umbilical cord-derived MSCs (hUC-MSCs) are popular in regenerative medicine due to their ability to be conveniently and minimally invasively acquired, their multi-lineage potential, immunoregulation capacity, and the minimal ethical issues (Nagamura-Inoue and Mukai, 2016). Normally, the blood-brain barrier prevents the penetration of MSCs, but it is believed that the integrity of the blood-brain barrier is impaired in response to injury or under neurodegenerative conditions, thereby facilitating the infiltration of MSCs into the brain. Accumulating evidence has shown that intravenously transplanted MSCs can penetrate the blood-brain barrier, dampen neural apoptosis, enhance neurogenesis, and improve learning and memory in AD mice (Mukai et al., 2018; Staff et al., 2019). MSCs have emerged as promising agents in combating AD. However, the underlying mechanisms remain unclear. Recent studies have suggested that MSCs can crosstalk with microglia and astrocytes. However, their role in regulating the efficacy of stem cell-based therapy in AD is restricted due to the low migration and survival rates of the transplanted cells under the adverse pathological microenvironment of the brain.

Optimization of MSC culture conditions by resveratrol can serve as a key strategy in improving MSC functioning in regenerative medicine (Hu and Li, 2019). Resveratrol is a stilbenoid found in various natural foods such as berries, grapes, peanuts, and blueberries. It has been widely studied and proven to be an anti-aging and anti-inflammatory agent, acting *via* SIRT1, NF-κB, and MAPK signaling (Shal et al., 2018), and is a particularly promising agent for the treatment of AD (Sawda et al., 2017). A previous experiment of ours showed that culturing with proper concentrations of resveratrol improved the proliferation and neural differentiation of hUC-MSCs *in vitro* (Wang et al., 2016). Other groups have also demonstrated that resveratrol pretreatment is safe, efficient, and low-cost, and pre-incubation of MSCs with resveratrol has yielded promising therapeutic effects on the treatment of acute kidney injury (Zhang et al., 2018), diabetic liver dysfunction, and pancreatic damage (Chen et al., 2019). Therefore, we speculate that resveratrol-primed MSCs are more resistant to chronic neuroinflammation in the brain of AD, and more efficient in treating AD.

In the current study, we compared the migratory ability of hUC-MSCs and resveratrol-preincubated hUC-MSCs (RES-MSCs) *in vitro* and in the hippocampus of AD mice, as well as their efficacy in rescuing pathological and behavioral deficiencies in AD mice. In addition, we investigated the hippocampal MAPK signaling pathways, which respond vigorously to various environmental stimuli, and play important roles in modulating inflammation and oxidative stress in the brain of AD mice (Franco et al., 2017; Lee and Kim, 2017). Our results showed that resveratrol enhanced the homing of MSCs into the hippocampus of AD mice, that RES-MSCs transplantation was a more effective approach for treating AD, and that the MAPK signaling pathway may be the underlying mechanism.

## Materials and Methods

### Preparation of hUC-MSCs

All procedures were performed in strict accordance with the National Institutes of Health guidelines for the Care and Use of Laboratory Animals and were approved by the Ethics Committees of the Zhengzhou University. Isolation and expansion of hUC-MSCs were performed according to our previous study (Ma et al., 2014). Passage 3 hUC-MSCs were cultured in DMEM/F12 media + 10% FBS with/without 2.5 μM resveratrol (Sigma-Adrich, St. Louis, MO, USA) for 6 days before transplantation. Surface marker characteristics were detected with flow cytometry.

### Transwell Migration Assay

Cell migration was assessed using 24-well plates containing Transwell inserts (8 μm, Corning, NewYork, NY, USA). Briefly, hUC-MSCs (1 × 10^5^) treated with or without 2.5 μM resveratrol were collected and suspended in 200 μl serum-free media and plated in the upper chamber. DMEM/F12 containing 10% FBS was added to the lower chamber, and, 24 h later, cells were fixed with methanol and stained with 0.1% crystal violet for 20 min. The upper cells were removed, and the cells which had migrated and accumulated on the other side of the transwell membrane were captured under bright field microscopy in five randomly selected fields and quantitatively represented as the mean count of stained cells per field. Experiments were independently repeated three times.

### Animals and Experimental Groups

Tg2576 Swedish transgenic AD mice which contain the human mutant transgene of APP695 (K670N/M671L) on a hamster prion promoter were used in this study. Age-matched C57BL/6 mice were used as wild-type (WT) controls. At 6 months, the mice were randomly divided into four experimental groups (15 mice/group), as shown in Table 1. This study was performed in strict accordance with the National Institutes of Health guidelines for the Care and Use of Laboratory Animals. No mouse presented any obvious signs of sickness or body weight change over the course of the study (Supplementary Figure S1). The experimental design of this research is shown in Figure 1.

**Table 1:** Experimental groups and treatment.

Group	Treatment
WT	C57BL6/J mice
AD	AD mice without any treatment
MSC	AD mice transplanted with hUC-MSCs*
RES-MSC	AD mice transplanted with resveratrol-preincubated hUC-MSCs*

*Cell transplantation: 1 × 10^6^ cells were collected and suspended in 200 μl of a saline solution and intravenously delivered to 6-month AD mice biweekly for 2 months.

**Figure 1:** Flowchart of the study design.

### Behavioral Studies

#### Morris Water Maze (MWM)

Behavioral studies were performed 4 weeks after stem cell transplantation. The MWM test was performed to evaluate spatial learning and memory of the mice, as previously described. The test was performed for seven consecutive days. During the training phase (the first 6 days), a platform (of a 10 cm diameter) was placed 1 cm below the surface of the water, and mice underwent four successive 60 s trials per day. The mice started from a different quadrant in each of the trials. The same quadrant start pattern was used across all trials. The latency for the mouse to find the platform was recorded. If a mouse did not find the platform in the first 60 s, it was gently guided towards the platform. Once a mouse was on the platform, it was allowed to sit on it for 30 s. The probe test was conducted on day seven. During this phase, the platform was removed and the mice then started from the quadrant opposite to the platform quadrant. The swimming path and the latency for the mouse to escape were recorded during the training. In addition, the number of times the mouse crossed the platform, the latency for the mouse to reach the platform location, and the time spent in the target quadrant was recorded by a video tracking system (Chengdu Taimeng Tech., Company Limited, China).

#### Y-maze Spontaneous Alternation Test (Y-maze)

The Y-maze spontaneous alternation test provides another assessment of working spatial memory (Sun et al., 2017). In short, in this test, the mouse was placed in the middle of the black-painted wood Y-maze (50 × 10 × 20 cm) and allowed to explore for 8 min. The Y-maze arms were thoroughly cleaned with 70% ethanol and allowed to dry to remove any residual odors after each test. The complete penetration of the hind paws of the mouse into the arm was counted as an arm entry. Consecutive entries into the three different arms were defined as exploration, and a spontaneous alternation rate was calculated as Alternation % = [Number of alternations/(Total arm entries − 2)] × 100. Mouse behaviors were recorded by a monitor right above the apparatus and analyzed using the ANY-maze video tracking software (Stoelting).

#### Novel Object Recognition Test (NOR)

The NOR test was used to evaluate the recognition memory of the mice based on their tendency towards novelty exploration. On the first day, the mice were placed in an open field apparatus (25 × 25 × 40 cm) in which they were allowed to habituate themselves for 5 min. The next day, two identical objects (round filter units, 33 mm diameter, 27 mm height) were placed in the central part of the test box, equally distant from the perimeter. The mice were then allowed to explore freely for 10 min (familiarization phase). On the third day, one clean familiar object and one clean novel object (plastic cone, 25 mm diameter, 30 mm height) were placed in the arena in which the two identical objects had been located during the familiarization phase, and the mice were allowed to explore for 5 min. To prevent any olfactory cues, the objects and the apparatus were cleaned with 70% ethanol after each trial. The time spent exploring each object was defined as directing the nose toward the object at a distance of no more than 2 cm or sniffing or touching the object with the nose. A single exploration of the object was set at a maximum period of 1.2 s, and any exploration longer than this time period was capped and recorded as 1.2 s. Mice with a total exploration time of less than 5 s in each test session were excluded from further analyses. The discrimination index was calculated as (time with novel object − time with familiar object)/(time with novel object + time with familiar object). Trials were tracked using an overhead monitor and analyzed using the ANY-maze video tracking software (Stoelting).

### Sample Collection

The mice were sacrificed after the behavioral study; they were anesthetized and fixed by cardiac perfusion with 4% paraformaldehyde. Then, brains were removed, post-fixed by incubation with 30% sucrose at 4°C until equilibrated. Sequential 20 μm coronal sections were taken on a cryostat (CM30 50S; Leica) and stored at −20°C for the experiment. For Western blotting and polymerase chain reaction (PCR), brains were immediately cut on the ice and the hippocampus was separated for further processing.

### Human-Specific DNA Assay

Total DNA was obtained from the hippocampus using a Tissue DNA kit (Lifefeng Biotechnology, China), and quantified with the NanoDrop 2000C spectrophotometer (Thermo Fisher Scientific, Waltham, MA, USA). The presence of human-specific DNA from migrated and survived hUC-MSCs was detected by PCR as previously described (Ehrhart et al., 2016).

### Immunofluorescence

The brain sections were prepared as described above and subjected to fluorescent immunostaining using the following primary antibody: anti-human nuclei antibody (MAB1281, 1:500, Millipore, Kankakee, IL, USA), glial fibrillary acidic protein (GFAP, 1:100, Proteintech, Rosemont, IL, USA), ionized calcium binding adapter molecule 1 (Iba1, 1:100, Proteintech, Rosemont, IL, USA), or 6E10 (1:1,000, BioLegend, San Diego, CA, USA). Negative controls were incubated with PBS instead of the primary antibody. The slides were then incubated in the secondary antibody: Cy3/FITC-conjugated anti-mouse/rabbit anti IgG (1:1,000, Molecular Probes, Eugene, OR, USA), followed by DAPI (1:1,000, Biotech, China) staining to visualize the cell nuclear. The sections were observed by microscopy (Olympus, Japan), and images of dentate gyrus areas of the hippocampus were visualized and captured using EC300 software. All images were captured using the same exposure times, contrast settings, and intensity for the measurement of fluorescence intensity. Fluorescence intensity, the area of positive immunofluorescence, or the number of immunofluorescent-positive cells were analyzed using ImageJ software. Data derived from three mice in each group and three slides for each mouse were quantified for further analyses.

### Quantitative Real-Time Polymerase Chain Reaction (qRT-PCR)

The mice hippocampus was homogenized in the ice, total RNA was extracted by Trizol reagent (Invitrogen, Waltham, MA, USA), and Complementary DNA (cDNA) was synthesized with Prime Script™ RT-PCR Kit (TaKaRa, Japan). qRT-PCR was performed by an ABI 7500 real-time PCR system (Thermo Fisher Scientific, Waltham, MA, USA) with SYBR Premix Ex Taq™ (Perfect Real Time, Japan). Relative expression of the target gene vs. Glyceraldehyde 3-phosphate dehydrogenase (GAPDH) was presented by 2^−ΔΔCt^. The primers sequences were shown in Table 2.

**Table 2:** Quantitative real-time polymerase chain reaction (qRT-PCR) primers sequences.

Gene	Sequence
TNF-α	5′-CACCACCATCAAGGACTCAA-3′ (F)
	5′-GAGACAGAGGCAACCTGACC-3′ (R)
IL-1β	5′-TGGGCTGGACTGTTTCTAATG-3′ (F)
	5′-GGTTTCTTGTGACCCTGAGC-3′ (R)
CD32	5′-AATCCTGCCGTTCCTACTGATC-3′ (F)
	5′-GTGTCACCGTGTCTTCCTTGAG-3′ (R)
iNOS	5′-TTGACCAGAGGACCCAGAGA-3′ (F)
	5′-AGCTGGTAGGTTCCTGTTGT-3′ (R)
IL-10	5′-AAATAAGAGCAAGGCAGTGG-3′ (F)
	5′-TCCAGCAGACTCAATACACAC-3′ (R)
CD206	5′-ACCCTGTATGCCTGTGATTC-3′(F)
	5′-ACTCTGTGCCCTTGATTCC-3′ (R)
Arg-1	5′-GGGAAAGCCAATGAAGAG-3′ (F)
	5′-AGGGGAGTGTTGATGTCAG-3′ (R)
IL-10	5′-GAAGACAATAACTGCACCCACT-3′ (F)
	5′-CTTAAAGTCCTGCATTAAGGAGTCG-3′ (R)
GAPDH	5′-GGTGAAGGTCGGTGTGAAC-3′ (F)
	5′-CCTTGACTGTGCCGTTGAA-3′ (R)

### Western Blotting

Hippocampal tissues were homogenized in an ice-cold lysis buffer containing protease inhibitors (YTHX Biotechnology). The lysate was centrifuged at 11,000 *g* at 4°C for 10 min followed by a BCA protein assay (Key GEN Biotech, China). An equal amount of protein was diluted by 4× gel-loading buffer before boiling for 5 min. The samples were then separated in SDS-PAGE gel and transferred to PVDF membranes (Sigma-Adrich, St. Louis, MO, USA). Membranes were blocked with 5% BSA in TBST for 2 h and incubated with primary antibodies overnight at 4°C: 6E10 (1:1,000, BioLegend, San Diego, CA, USA), microtubule-associated protein tau (MAPT, 1:1,000, Shenggong, China), and phospho-Ser396/Thr231/Ser202 MAPT (1:1,000, Shenggong, China), ERK1/2 (1:1,000; Cell Signaling Technology, Danvers, MA, USA), p-ERK (1:1,000, Cell Signaling Technology, Danvers, MA, USA), p38 (1:1,000, Santa Cruz Biotechnology, Dallas, TX, USA), p-p38 (1:1,000, Santa Cruz Biotechnology, Dallas, TX, USA), Jun N-terminal kinases (JNK; 1:1,000; Santa Cruz Biotechnology, Dallas, TX, USA), p-JNK (1:1,000, Santa Cruz Biotechnology, Dallas, TX, USA), washed three times in TBST for 10 min each time, followed by incubation with HRP-conjugated secondary antibody for 1 h at room temperature, and washed three times. Finally, proteins were visualized by enhanced chemiluminescence reagents. ImageJ software was used to semi-quantify the relative expression of target proteins vs. β-actin.

### Measurement of Antioxidant Capacity

After sacrifice, the brains of the mice were quickly collected on the ice, washed with pre-cooled 0.9% saline solution, and weighed. Saline solution was added to make a 10% brain homogenate and centrifuged at 10,000 *g* for 10 min at 4°C. The supernatant of the brain homogenate was used to determine the levels of Superoxide dismutase (SOD), Glutathione peroxidase (GSH-Px), catalase (CAT), and malondialdehyde (MDA) using commercial kits purchased according to the manufacturer’s instructions, as previously described (Samad et al., 2019).

### Statistical Analysis

The data were expressed as mean ± SEM and statistically analyzed using GraphPad Prism 8 or SPSS 22. Data were tested for normality and its Gaussian distribution was verified. A Student’s *t*-test was used to compare the two experimental groups in the cell migration experiments in Figures 2, 3, and explore preference for two objects in Figures 4G,H Multi-group comparisons were processed by one-way ANOVA followed by Bonferroni’s *post hoc* correction. This was used to analyze the data obtained from the probe trial test of MWM (Figures 4C–E), Y-maze (Figure 4F), discrimination index in NOR (Figure 4I), and data of immunofluorescence, qRT-PCR, Western blotting, SOD, GSH-Px, CAT, and MDA (Figures 5–9). Repeated measure ANOVA was used to analyze the latency to the platform in the 6-day spatial acquisition test of MWM (Figure 4B). *p* < 0.05 was considered statistically significant. Data shown were representative of at least three independent experiments.

**Figure 2:** Effect of resveratrol on the migration of hUC-MSCs. **(A)** The hUC-MSCs that migrated to the bottom of the transwell insert were stained with crystal violet. Scale bars = 50 μm. **(B)** Graphical representation of the quantification of migrated cells. The number of migrated cells was counted using five random fields per well. Each experiment was repeated thrice (*n* = 15). Data were presented as mean ± SEM (*t*-test: ****indicates *p* < 0.0001; MSC vs. RES-MSC). MSC, human umbilical cord-derived mesenchymal stem cells; RES-MSC, human umbilical cord-derived mesenchymal stem cells pretreated with 2.5 μM resveratrol for 6 days; SEM, standard error of mean.

**Figure 3:** Resveratrol enhanced the engraftment of hUC-MSCs in the brain of Alzheimer’s disease (AD) mice. The hUC-MSCs were identified in the hippocampal sections of AD mice, 6 weeks after completion of cell transplantation, by their immunoreactivity to the human anti-nuclei antibody, MAB1281. **(A)** Representative immunofluorescent images of MAB1281+ cells in the hippocampus. Scale bar = 50 μm. **(B)** Quantitative analysis of MAB1281+ cells in the hippocampus. Data were acquired from three mice in each group and from three slides of each mouse hippocampus (*n* = 9) and were presented as mean ± SEM (*t*-test: ****indicate *p* < 0.0001; MSC vs. RES-MSC). **(C)** Results of polymerase chain reaction (PCR) results of human-specific DNA in the mouse hippocampus. **(D)** Quantification of human-specific DNA in different groups. Data were acquired from three mice in each group and each experiment was repeated thrice (*n* = 9) and were expressed as mean ± SEM (*t*-test: ****indicate *p* < 0.0001; MSC vs. RES-MSC). MSC, mice treated with mesenchymal stem cells; RES-MSC, mice treated with resveratrol pre-incubated mesenchymal stem cells.

**Figure 4:** MSCs and RES-MSCs improved the cognitive functions of AD mice. **(A)** The swimming path during the training period of morris water maze (MWM). **(B)** The learning curve during the training period of MWM (Repeated ANOVA, *p < 0.05, **p < 0.01, ***p < 0.001, ****p < 0.0001 vs. AD). **(C)** The frequency of crossing the hidden platform (ANOVA plus Bonferroni, wild-type (WT) vs. AD *p* < 0.0001, MSC vs. AD *p* = 0.0355, RES-MSC vs. AD *p* < 0.0001, MSC vs. RES-MSC *p* = 0.0355). **(D)** The percentage of time spent in the target quadrant (ANOVA plus Bonferroni: WT vs. AD *p* < 0.0001, MSC vs. AD *p* = 0.0028, RES-MSC vs. AD *p* < 0.0001, MSC vs. RES-MSC *p* = 0.012), and **(E)** the escape latency during the probe trial of MWM (ANOVA with Bonferroni correction, WT vs. AD, *p* < 0.0001; MSC vs. AD, *p* < 0.0001; RES-MSC vs. AD, *p* < 0.0001; MSC vs. RES-MSC, *p* < 0.0001). **(F)** Alternation rates in the Y-maze test (ANOVA plus Bonferroni: WT vs. AD *p* < 0.0001, MSC vs. AD *p* = 0.0023, RES-MSC vs. AD *p* < 0.0001, MSC vs. RES-MSC *p* = 0.0369). **(G)** Exploration times for two identical objects during the training session of the Y-maze test (*t*-test, *p* > 0.05). **(H)** Exploration time for familiar or novel object during the test session (*t*-test, WT: *p* = 0.0002. AD: *p* = 0.4784. MSC: *p* = 0.0167. RES-MSC *p* = 0.0007). **(I)** Discrimination index were measured in the NOR test (ANOVA plus Bonferroni, WT vs. AD *p* < 0.0001, MSC vs. AD *p* = 0.1854, RES-MSC vs. AD *p* < 0.0001, MSC vs. RES-MSC *p* = 0.0464). The data were collected from 15 mice per group (*n* = 15), and expressed as mean ± SEM. *p < 0.05, **p < 0.01, ***p < 0.001, ****p < 0.0001.

**Figure 5:** MSCs and RES-MSCs regulated the expression of APP in mouse hippocampus. **(A)** Representative immunohistochemical images and** (B)** the relative fluorescence intensity of APP immunostaining in the hippocampus. Scale bar = 50 μm. The area of positive immunofluorescence was analyzed. Data were derived from three mice in each group and from three sections of each mouse (*n* = 9). Results were expressed as mean ± SEM and analyzed by ANOVA plus Bonferroni (WT vs. AD *p* < 0.0001, MSC vs. AD *p* < 0.0001, RES-MSC vs. AD *p* < 0.0001, MSC vs. RES-MSC *p* < 0.0001). **(C)** Representative images of Western blotting of APP **(D)** The gray values of the Western blotting of APP were analyzed from three mice in each group and from three independent experiments from each mouse (*n* = 9). Results were expressed as mean ± SEM (ANOVA plus Bonferroni: WT vs. AD *p* < 0.0001, MSC vs. AD *p* = 0.1854, RES-MSC vs. AD *p* < 0.0001, MSC vs. RES-MSC *p* = 0.0443). *p < 0.05, ****p < 0.0001.

**Figure 6:** MSCs and RES-MSCs down-regulated the phosphorylation of tau in the hippocampus. **(A)** Representative images of Western Blotting of total MAPT and phospho-Ser396/Thr231/Ser202 MAPT. **(B)** The gray values were analyzed based on values from three mice in each group and from three independent experiment from each mouse (*n* = 9). Results were expressed as mean ± SEM. **p < 0.01, ***p < 0.001, ****p < 0.0001 (ANOVA plus Bonferroni: p-Ser396 MAPT: WT vs. AD *p* < 0.0001, MSC vs. AD *p* < 0.0001, RES-MSC vs. AD *p* < 0.0001, MSC vs. RES-MSC *p* = 0.0002. p-Thr231 MAPT: WT vs. AD *p* < 0.0001, MSC vs. AD *p* = 0.0004, RES-MSC vs. AD *p* < 0.0001, MSC vs. RES-MSC *p* = 0.002. p-Ser202 MAPT: WT vs. AD *p* < 0.0001, MSC vs. AD *p* < 0.0001, RES-MSC vs. AD *p* < 0.0001, MSC vs. RES-MSC *p* = 0.0026. MAPT: WT vs. AD *p* = 0.09981, MSC vs. AD *p* > 0.9999, RES-MSC vs. AD *p* > 0.9999, MSC vs. RES-MSC *p* > 0.9999).

**Figure 7:** MSCs or RES-MSCs inhibited oxidative stress in the hippocampus. Measurement of antioxidant molecules **(A)** SOD, **(B)** GSH-Px, and **(C)** CAT, and the level of **(D)** MDA in the hippocampus among the experimental groups. Data were collected from 15 mice per group (*n* = 15). Results were expressed as mean ± SEM. *p < 0.05, **p < 0.01, ***p < 0.001, ****p < 0.0001 (ANOVA plus Bonferroni: SOD: WT vs. AD *p* < 0.0001, MSC vs. AD *p* < 0.0001, RES-MSC vs. AD *p* < 0.0001, MSC vs. RES-MSC *p* = 0.0191. GSH-Px: WT vs. AD *p* < 0.0001, MSC vs. AD *p* < 0.0001, RES-MSC vs. AD *p* = 0.0003, MSC vs. RES-MSC *p* = 0.0062. CAT: WT vs. AD *p* < 0.0001, MSC vs. AD *p* < 0.0001, RES-MSC vs. AD *p* < 0.0001, MSC vs. RES-MSC *p* = 0.0003. MDA: WT vs. AD *p* < 0.0001, MSC vs. AD *p* < 0.0001, RES-MSC vs. AD *p* < 0.0001, MSC vs. RES-MSC *p* = 0.0136).

**Figure 8:** MSCs or RES-MSCs regulated astrocyte- and microglia-mediated inflammation in the hippocampus of AD mice. Representative immunostained images of GFAP^+^ astrocyte **(A)** and Iba1^+^ microglia **(B)**. Scale bar = 50 μm. Semi-quantitative analysis of the immunopositive fluorescent intensity of GFAP **(C)** and Iba1 **(D)**. Intensities of immunofluorescence were analyzed from three mice in each group and from three section from each mouse hippocampus (*n* = 9). Results were expressed as mean ± SEM. *p < 0.05, **p < 0.01, ***p < 0.001, ****p < 0.0001 (ANOVA plus Bonferroni: GFAP: WT vs. AD *p* < 0.0001, MSC vs. AD *p* = 0.0369, RES-MSC vs. AD *p* < 0.0042, MSC vs. RES-MSC *p* = 0.0033. Iba1: WT vs. AD *p* < 0.0001, MSC vs. AD *p* = 0.0007, RES-MSC vs. AD *p* < 0.0001, MSC vs. RES-MSC *p* = 0.0042). **(E)** qRT-PCR results indicating the relative expression of microglia M1 phenotype markers (TNF-α, IL-1β, CD32, and iNOS) and **(F)** M2 phenotype marker (IL-10, CD206, Arg-1, and Ym1/2) in the hippocampus of the mice. Values were obtained from three mice of each group and from the results of three independent experiments from each mouse (*n* = 9). The expression of genes were normalized to that of GAPDH and quantified relative to that of the WT mice. Results were expressed as mean ± SEM. *p < 0.05, **p < 0.01, ***p < 0.001, ****p < 0.0001 (ANOVA plus Bonferroni: *p < 0.05, **p < 0.01, ***p < 0.001, ****p < 0.0001. TNF-α: WT vs. AD *p* < 0.0001, MSC vs. AD *p* = 0.0163, RES-MSC vs. AD *p* < 0.0001, MSC vs. RES-MSC *p* = 0.0152. IL-1β: WT vs. AD *p* < 0.0001, MSC vs. AD *p* = 0.0247, RES-MSC vs. AD *p* < 0.0001, MSC vs. RES-MSC *p* = 0.0422. CD32: WT vs. AD *p* < 0.0001, MSC vs. AD *p* = 0.0139, RES-MSC vs. AD *p* < 0.0001, MSC vs. RES-MSC *p* = 0.0092. iNOS: WT vs. AD *p* < 0.0001, MSC vs. AD *p* = 0.0013, RES-MSC vs. AD *p* < 0.0001, MSC vs. RES-MSC *p* = 0.0032. IL-10: WT vs. AD *p* < 0.0001, MSC vs. AD *p* < 0.0001, RES-MSC vs. AD *p* < 0.0001, MSC vs. RES-MSC *p* = 0.0227. CD206: WT vs. AD *p* < 0.0001, MSC vs. AD *p* = 0.0028, RES-MSC vs. AD *p* < 0.0001, MSC vs. RES-MSC *p* = 0.0003. Arg-1: WT vs. AD *p* < 0.0001, MSC vs. AD *p* < 0.0001, RES-MSC vs. AD *p* < 0.0001, MSC vs. RES-MSC *p* < 0.0001. Ym1/2: WT vs. AD *p* < 0.0001, MSC vs. AD *p* = 0.0002, RES-MSC vs. AD *p* < 0.0001, MSC vs. RES-MSC *p* = 0.0117).

**Figure 9:** MSCs and RES-MSCs regulated MAPK signaling in the hippocampus of AD mice. **(A)** Representative images of Western blotting of p38, JNK, ERK, and phosphorylated p38, JNK, and ERK.** (B)** Relative expression of p-p38/total p38, p-JNK/total JNK, and p-ERK/total ERK in mice hippocampus. Analysis of the gray values from Western blotting obtained for three mice from each group and from three independent experiments from each *mouse* (*n* = 9). Results were expressed as mean ± SEM. *p < 0.05, **p < 0.01, ***p < 0.001, ****p < 0.0001 (ANOVA plus Bonferroni: p-p38/p38: WT vs. AD *p* < 0.0001, MSC vs. AD *p* = 0.0043, RES-MSC vs. AD *p* < 0.0001, MSC vs. RES-MSC *p* = 0.0003. p-JNK/JNK: WT vs. AD *p* = 0.0002, MSC vs. AD *p* = 0.0171, RES-MSC vs. AD *p* = 0.0007, MSC vs. RES-MSC *p* = 0.0186. p-ERK/ERK: WT vs. AD *p* < 0.0001, MSC vs. AD *p* = 0.0097, RES-MSC vs. AD *p* = 0.0001, MSC vs. RES-MSC *p* = 0.0135).

## Results

### Resveratrol Promoted the Migration of hUC-MSCs *in vitro*

RES-MSCs retained the spindle-shaped morphology and expressed the classical surface markers of hUC-MSCs. Resveratrol promoted the migration of hUC-MSCs as evidenced by the results of the Transwell assay (Figures 2A,B).

### Resveratrol Pretreatment Facilitate the Survival and Homing of hUC-MSCs in the Hippocampus

The survival and homing of hUC-MSCs in the brain of AD mice were detected 6 weeks after completion of cell transplantation. We found that RES-MSCs significantly improved the ability to migrate into the hippocampus, as demonstrated by immunofluorescence with human nuclei antibody (MAB1281; Figures 3A,B) and PCR of human-specific DNA (Figures 3C,D).

### Resveratrol Pretreatment Improved the Effect of hUC-MSCs on Cognitive Retrieval for AD Mice

The MWM test, Y-maze test, and NOR test were performed 4 weeks after MSCs/RES-MSCs transplantation to evaluate the learning and memory ability of 9-month-old mice. AD mice exhibited a compromised learning and memory capacity compared to their WT counterparts, and hUC-MSCs transplantation improved the learning of AD mice as evidenced by their swimming path (Figure 4A) and their learning curve (Figure 4B) during training in MWM test. Results revealed that, during the 6-day training phase, compared to the WT mice, AD mice exhibited significantly longer escape latencies. However, when subjected to MSCs, their escape latency was significantly shorter, indicating an enhanced learning ability. In addition, significantly increased frequencies of crossing the platform location (Figure 4C), a longer time spent in the target quadrant (Figure 4D), and shorter escape latencies (Figure 4E) were shown in the MSC group in the probe test of the MWM, indicating an improved memory. Moreover, the learning and memory of the AD mice could be further enhanced by RES-MSCs.

The Y-maze test was another way of assessing working memory. It was demonstrated that the alternation rate was significantly increased in groups of MSCs and RES-MSCs compared to AD mice (Figure 4F), and significantly increased in the RES-MSCs group compared to the MSCs group.

In terms of the NOR, previous studies performed in our laboratory have demonstrated that mice did not display a spontaneous preference for any of the different objects used in the current study (Supplementary Figure S2). There was no difference between the exploration times of the two identical objects during the familiarization phase (Figure 4G). Mice tend to explore novel objects (Figure 4H); however, the discrimination index was reduced in AD mice, and hUC-MSCs treatment could significantly restore memory and increased the discrimination index (Figure 4I). This was further increased by RES-MSCs treatment.

### MSCs and RES-MSCs Reduced APP Expression in the Hippocampus

Transgenic AD mice overexpressed amyloid protein precursor (APP), as demonstrated by immunofluorescence and Western Blotting with a 6E10 antibody. However, this was significantly reduced by hUC-MSCs transplantation, and even more obvious changes were demonstrated in the RES-MSCs group (Figures 5A–D).

### MSCs and RES-MSCs Down-Regulated the Phosphorylation of Tau in the Hippocampus of AD Mice

Western Blotting of phospho-Ser396/Thr231/Ser202 MAPT showed that hUC-MSCs transplantation inhibited the hyperphosphorylation of Tau in AD mice, and RES-MSCs enhanced these effects of hUC-MSCs (Figures 6A,B).

### MSCs and RES-MSCs Inhibited Oxidative Stress in the Hippocampus of AD Mice

Oxidative stress was intimately associated with the pathology of AD. We found that hUC-MSCs transplantation protects the brain from oxidative stress, as evidenced by a significant increase in vital antioxidant enzymes, SOD, GSH-Px, and CAT activity, and a reduction in MDA, a neurotoxic product of lipid peroxidation. Furthermore, these beneficial effects were remarkably enhanced by RES-MSCs transplantation (Figures 7A–D).

### MSCs and RES-MSCs Down-Regulated the Activation of Astrocytes and Microglia in the Hippocampus and Converted Microglia Polarization From M1 to M2

Activated astrocytes and microglia were detected by GFAP and Iba1, respectively. We found that GFAP^+^ cells and Iba1^+^ cells were significantly increased in AD mice and reduced after MSCs or RES-MSCs treatments (Figures 8A–D). Moreover, expression levels of M1 phenotypic markers (TNF-α, IL-1β, CD32, and iNOS) in the hippocampus were downregulated and expression levels of M2 phenotypic markers (IL-10, CD206, Arg-1, and Ym1/2) were up-regulated by hUC-MSCs, most significantly in the RES-MSCs group (Figures 8E,F).

### MSCs and RES-MSCs Repressed the MAPK Signaling Pathway in the Hippocampus of AD Mice

Western blotting revealed that the phosphorylation levels of p38, JNK, and ERK in the hippocampus of AD mice were increased compared with those of WT mice, which were down-regulated by hUC-MSCs transplantation and further reduced in the RES-MSCs group (Figures 9A,B).

## Discussion

AD is a complicated neurodegenerative disease clinically characterized by a progressive loss of cognition (Derakhshankhah et al., 2020). The pathological hallmarks of the disease include extracellular aggregates of Aβ and tau-associated pathology. Current therapeutic agents are not only inadequate to suppress the progression of AD pathogenesis but also produce deleterious side effects. Given the aging population worldwide, searching for novel therapies for AD is an urgent priority (Sawda et al., 2017). Stem cells, especially MSCs, have great potential to delay the onset or progression of AD. However, low migration, survival, and neural differentiation rates are the key factors in determining therapeutic efficacy in translational studies (Chakari-Khiavi et al., 2019). Accumulating evidence has demonstrated that the preconditioning of stem cells prior to transplantation could promote cell survival and efficacy (Pourjafar et al., 2017; Hu and Li, 2018; Esmaeilzade et al., 2019). Resveratrol, an activator of SIRT1, is an antiaging regent which could protect cells against oxidative stress and nutrient stressors (Gomes et al., 2018). The current study was designed to improve MSC-based therapy for AD by pre-incubating hUC-MSCs with resveratrol.

This study’s results revealed that preconditioning with resveratrol increased the hUC-MSCs number in the DG of AD mice. The DG niche in the hippocampus was the hub for neurogenesis, learning, and memory, yet was also an area more susceptible to deterioration under aging and AD (Lazarov and Marr, 2010). MSCs tend to home to injury areas by inflammatory factors or other signals, thereby, we focused on the migration of stem cells into the DG of the hippocampus, and cellular and molecular changes in this area. Our previous *in vitro* study has revealed that (Wang et al., 2016, 2018) resveratrol could enhance cell viability, proliferation, and neural differentiation, and inhibit the senescence of hUC-MSCs *via* SIRT1 signaling. Furthermore, the present study showed that resveratrol facilitated the migration of hUC-MSCs *in vivo* and *in vitro*, resulting in an enhancement of engraftment of hUC-MSCs in the DG of AD mice.

It was demonstrated in the current study that resveratrol-exposed hUC-MSCs could, to a larger degree, dampen Aβ accumulation, and alleviate tau hyperphosphorylation in the DG of AD mice. The DG plays an important role in the acquisition of new information, memory formation, and mediating various mnemonic processing, including conjunctive encoding of multiple sensory inputs to determine spatial representations, object recognition, pattern separation, short-term memory, and remote time-based memory (Kesner, 2018). An alleviated microenvironment in the DG contributed to the behavioral improvement in MWM, Y-maze, and NOR in the present study.

We also found that hUC-MSCs could reduce oxidative stress in the brains of AD mice. Some researchers demonstrated that extracellular vesicles secreted by MSCs (MSC-MVs) carried endogenous antioxidant enzymes (e.g., catalase) that endowed ROS scavenging activity (de Godoy et al., 2018). MSC-MVs were able to prevent the expression of PTGS2 transcripts and reduce iNOS enzymes and NO injury (Jaimes et al., 2017). Moreover, ROS production in MSCs could be inhibited by resveratrol (Zhou et al., 2019). Therefore, resveratrol-treated hUC-MSCs showed better antioxidant effects.

To further explore the pathological change after hUC-MSCs transplantation, we studied neuro-inflammation in DG. A previous study demonstrated that the hUC-MSCs conditioned medium promoted the phagocytosis of Aβ25–35 by BV2 microglial cells *in vitro* and upregulated the expression of neprilysin and insulin-degrading enzymes, major proteases which cleave Aβ plaques (Xu et al., 2018). Aβ deposition is recognized as the main culprit for the pathological cascade of AD. Increasing evidence has demonstrated that accumulated Aβ in AD causes microglial activation and astrocyte recruitment, thereby generating free radicals, nitric oxide, and pro-inflammatory cytokines (Cai et al., 2014; Das and Chinnathambi, 2019). Activated inflammation, in turn, could induce BACE-1 expression, facilitate Aβ deposition, and exacerbate neurofibrillary tangles, leading to a vicious cycle in which neurons are gradually damaged (Lee et al., 2008; Heneka et al., 2015; Kinney et al., 2018). Inflammation is the core driver of this vicious cycle of AD pathogenesis. Therefore, in the current study, we sought to investigate the effects of hUC-MSCs and RES-MSCs on microglia and astrocyte-mediated neuroinflammation.

It is known that microglia are the primary inflammatory cells in the brain. However, they have a dual role which remains contentious. Microglia can exhibit two phenotypes: M1 (pro-inflammatory) and M2 (anti-inflammatory) (Yao and Zu, 2019). Microglial cells are able to remove Aβ deposits in the early stages of a lesion but fail to do so as the disease progresses. Instead, they become chronically activated and release pro-inflammatory factors and ROS, leading to the disruption of the blood-brain barrier, synapse loss, and neurotoxicity (Sarlus and Heneka, 2017). Our study revealed a decrease in the number of Iba1^+^ microglial cells in the hippocampus of AD mice after hUC-MSCs transplantation. Besides, transplanted hUC-MSCs modulated microglial polarization, as evidenced by the down-regulated expression of M1 phenotypic markers (TNF-α, IL-1β, CD32, and iNOS) and upregulated M2 phenotypic markers (IL-10, CD206, Arg-1, and Ym1/2). It was recognized that MSCs could secrete a panel of cytokines, chemokines, growth factors, and metabolites, among which, TGF-β and CX3CR1 have been reported to exert important roles in M1 phenotype shift to the protective M2 microglia (Noh et al., 2016; Barati et al., 2019). Furthermore, RES-MSCs facilitated the polarization of microglial cells from an M1 to an M2 status, demonstrating that microglia-mediated neuroinflammation was further inhibited.

Astrocytes, the most abundant glial subtype in the CNS, also play an important but controversial role in AD. Astrocytes produce a wide array of inflammatory cytokines that can be either beneficial or detrimental (Colombo and Farina, 2016). Söllvander et al. (2016) proposed that excessive phagocytosis of Aβ resulted in incomplete digestion, accumulation, and spread of toxic Aβ species, eventually leading to astrocytic defects and neuronal apoptosis, even though astrocytes mediate the degradation of amyloid plaques. Also, astrocytes could produce Aβ under certain conditions (Zhao et al., 2011), pointing to a complicated role of astrocytes in the progression of AD. In line with a previous study (Nagele et al., 2003), we found excessive astrogliosis in the hippocampus of AD mice, which may lead to glial scarring. However, the number of GFAP^+^ astrocytes was decreased after hUC-MSCs transplantation and reduced to an even larger extent in the RES-MSCs group. Therefore, our results clearly demonstrated the positive role of stem cell therapy in reducing neuroinflammation and gliosis, which may be the result of rejuvenating cell activity in astrocytes and microglia.

To explore the underlying molecular mechanisms, we assessed the MAPK signaling pathway, which plays distinct roles in Aβ deposition, tau phosphorylation, and synaptic dysfunction, as well as microglia and astrocyte-mediated neuroinflammation and impairment (Lee and Kim, 2017). Many researchers have attempted to inhibit MAPK signaling in glial cells to treat AD (Mehan et al., 2011; Yamamoto et al., 2016; Yang et al., 2017). In addition to chemical inhibitors, Jaimes et al. (2017) reported that MSCs could modulate microglia-mediated inflammatory responses by inhibiting the phosphorylation of the MAPK family members ERK1/2, p38, and JNK. Huang et al. (2015) also reported that paracrine factors secreted by MSCs protected astrocytes from oxygen-glucose deprivation/reperfusion-induced injury, and attenuated apoptosis and GFAP overexpression *via* suppressing p38 MAPK and JNK. Consistent with these *in vitro* results, we found that the activated MAPK signaling cascades in the hippocampus of AD mice were significantly inhibited by hUC-MSCs and RES-MSCs transplantation, as shown by the decreased phosphorylation of ERK, p38, and JNK, important functional molecules of the MAPK family.

Previous literature has demonstrated that MSCs could regulate gene expression by paracrine and delivery of mRNAs, miRNA, noncoding RNAs, or transcription factors to target cells (Qiu et al., 2018; Elia et al., 2019). For instance, the miR-21 secreted by MSCs could dampen the activation of NF-κB, c-Jun/AP1, and STAT3 signaling, which were relevant in the neuro-inflammation in AD (Das et al., 2014; Cui et al., 2018). We conclude that hUC-MSCs and RES-MSCs exert an anti-inflammation effect in AD at least partially through the inhibition of MAPK activation. And we speculate that the MAPK signaling in the AD brain may also be regulated by specific mRNAs, miRNA, noncoding RNAs, or transcription factors secreted by hUC-MSCs. However, further study is required to reveal how the MAPK cascade is disrupted by transplanted hUC-MSCs and RES-MSCs in AD mice.

## Conclusion

This study revealed that hUC-MSCs could reverse the pathological and cognitive decline by modulating microglia and astrocyte-mediated inflammation in the hippocampus of AD mice, with MAPK as the key signaling mechanism. Furthermore, resveratrol preincubation facilitated the migration of hUC-MSCs in the hippocampus of AD mice, and positively contributed to the outcomes of hUC-MSCs in the context of AD treatment. Optimizing the culture conditions of hUC-MSCs by resveratrol can serve as an efficient strategy in improving the function of the transplanted cells in AD mice. This study will promote the clinical applicability of RES-MSCs for the management of AD. However, it should be noted that the distribution and effects of hUC-MSCs in the brain may vary depending on the type of disease model and specific time during the migration of the cells. It is interesting to unveil more detailed pathological processes and time-dependent responses to the hUC-MSCs treatment in different brain regions of AD in future studies.

## Data Availability Statement

The datasets generated for this study are available on request to the corresponding author.

## Ethics Statement

The animal study was reviewed and approved by the Ethics Committees of the Zhengzhou University.

## Author Contributions

FG, RG, and BY conceived the project, interpreted the data, edited the manuscript, and provided financial support. XW and JW designed the study, performed the experiments, collected and analyzed the data, and drafted the manuscript. SM, YX, HL, MY, YZ, and GY contributed to the design and implementation of the research, and editing. All authors approved the final draft of the article.

## Conflict of Interest

The authors declare that the research was conducted in the absence of any commercial or financial relationships that could be construed as a potential conflict of interest.

## Supplementary Material

FIGURE S1 Body weights of the experimental mice. There is no significant difference in the body weight of mice in each experimental group.

FIGURE S2 The AD mice explore each object in the NOR equally.
